The article "Height, Socioeconomic and Subjective Well-Being Factors among U.S. Women, Ages 49–79" was published in 2014. Journal: PLoS One.

# Height, Socioeconomic and Subjective Well-Being Factors among U.S. Women, Ages 49–79

**DOI:** 10.1371/journal.pone.0096061

**Published:** 2014-06-04

**Authors:** Grace Wyshak

**Affiliations:** Harvard Medical School, Department of Psychiatry and Harvard School of Public Health, Departments of Biostatistics and Global Health and Population, Boston, Massachusetts, United States of America; Federal University of Rio de Janeiro, Brazil

## Abstract

**Background:**

A vast literature has associated height with numerous factors, including biological, psychological, socioeconomic, anthropologic, genetic, environmental, and ecologic, among others. The aim of this study is to examine, among U.S. women, height factors focusing on health, income, education, occupation, social activities, religiosity and subjective well-being.

**Methods/Findings:**

Data are from the Women's Health Initiative (WHI) Observational Study. Participants are 93,676 relatively healthy women ages 49–79; 83% of whom are White, 17% Non-White. Statistical analyses included descriptive statistics, chi-square and multivariable covariance analyses.

The mean height of the total sample is 63.67 inches. White women are significantly taller than Non-White women, mean heights 63.68 vs. 63.63 inches (p = 0.0333).

Among both Non-White and White women height is associated with s**ocial** behavior, i.e. attendance at clubs/lodges/groups. Women who reported attendance ‘once a week or more often’ were taller than those who reported ‘none’ and ‘once to 3 times a month’. Means in inches are respectively for: White women–63.73 vs. 63.67 and 63.73 vs. 63.67, p = 0.0027. p = 0.0298; Non-White women: 63.77 vs. 63.61 and 63.77 vs. 63.60, p = 0.0050, P = 0.0094. In both White and Non-White women, income, education and subjective well-being were not associated with height.

However, other factors differed by race/ethnicity. Taller White women hold or have held managerial/professional jobs–yes vs. no–63.70 vs. 63.66 inches; P = 0.036; and given ‘a little’ strength and comfort from religion’ compared to ‘none’ and ‘a great deal’, 63.73 vs. 63.66 P = 0.0418 and 63.73 vs. 63.67, P = 0.0130. Taller Non-White women had better health—excellent or very good vs. good, fair or poor–63.70 vs. 63.59, P = 0.0116.

**Conclusions:**

Further research in diverse populations is suggested by the new findings: being taller is associated with social activities –frequent attendance clubs/lodges/groups”, and with ‘a little’ vs. ‘none’ or ‘great deal’ of strength and comfort from religion.

## Introduction

Height has been a subject of interest, discussion and analyses as early as biblical times. For example, “In the first book of Samuel we read the account of Saul being selected king. While Saul's qualifications for the job were not described in any detail, there is one attribute specifically mentioned: he was tall.” [1]. In the twenty first century (2012), Ozaltin outlined six mechanisms that account for the association between height and adult outcomes—genetic, biological, psychosocial, biomechanical, epigenetic, confounding or endogeniety [2]. Steckel examined the unique and valuable contributions of four biological measures—life expectancy, morbidity, stature, and certain features of skeletal remains—to understand levels and changes in human well-being [3]. In 2009 he notes the increasing interest in height (stature): “Since 1995 approximately 325 publications on stature have appeared in the social sciences, which is more than a four-fold increase in the rate of production relative to the period 1977–1994” [4].

The body of literature on height is global, vast and increasing [4]. Cited here are a selected number of papers that relate to height and a broad range of factors including: genetics, early life development, nutrition, biology, socioeconomic factors [5]–[9], [14]–[24], [26]–[29]; medical conditions include infection [6], coronary heart diseases [5], cardiorespiratory disease and cancer mortality [9], dementia [28]; economic factors are income [7], [10], [15], wages [16], [21], wealth [25]; education [8], [10]; cognitive skills [7], [13]; occupation/workplace, [11], [12], [15], [20], [21], [29]; psychological factors—success [1], [12],choices [13]; for women, reproduction [22] marriage [24], gender inequality [18]; comparisons at the country level [7], [8], [18], [25]. Height, income and education are the primary variables analyzed from The Gallup-Healthways Well-Being Index daily poll of the US population [10].

The general conclusion from the literature cited is: Taller is associated with favorable early environment, nutrition, medical conditions, health, income and education in both men and women. However, there are exceptions: i) the significant association of height and income were not found [14], [16]; ii) taller women, but not men, had more upward mobility in both white and blue collar occupations [16]; iii) upward mobility was not associated with health [16]. By analyzing data from a survey of a diverse group of relatively healthy U.S. women, ages 49–79, this study adds to the substantial knowledge base on height and other outcomes. It suggests areas for further research, particularly by its new findings and insights on height with its associations with religiosity and with social behavior (here denoted by attendance at clubs)—two constructs, to my knowledge not heretofore cited in the literature or among the six mechanisms, outlined by Ozaltin, that account for the association between height and adult outcomes of height [2].

## Materials and Methods

My paper is data from the WHI Baseline Data Set of 10/16/2003, Women's Health Initiative Observational Study, provided by the National Heart, Lung and Blood Institute; the data set was converted to a SAS file in 2013. This study examines the association between height and some of the factors cited in the literature such as demographics—age, gender, ethnicity, income, education, occupation–health, social, subjective well-being, among relatively healthy women, 49–79 years of age, who participated in the Women's Health Initiative's Observational Study (WHI OS). Its main purpose is to assess a wide variety of important clinical and public health issues. Enrollment was conducted at 40 centers throughout the US. The justification for the WHI study is: “There is a general recognition that few older women have been studied longitudinally and that major questions about prediction of chronic disease in postmenopausal women remain.” “Participants in the observational study were women aged 49–79 (mean age 63.62, standard deviation, 7.37), who were ineligible or unwilling to participate in the clinical trial component or were recruited through a direct invitation for screening into the observational study.” “Many potential participants in the clinical trial component of the study were already undertaking a low fat diet or were using hormone replacement therapy and therefore were excluded or declined to participate clinical trial component. These participants were then enrolled into the observational study. Previous research has demonstrated that at the time of WHI enrollment, women undertaking hormone replacement therapy and/or low fat diets generally had healthier lifestyles than those not possessing these behaviors. The effect of the selection process was that women enrolled in the observational study tended to have healthier lifestyles compared to those enrolled in the clinical trial.” The data set consists of 2022 variables including demographics, eligibility for selection, personal information, medical history, reproductive history, family history, personal habits, thoughts and feeling, and other areas. Participants are 93,676 women—83% (78,013) White, 17% Non-White– 8% Black (7,639), 4% Hispanic (2,623); the remaining 5% Asian/Pacific Islander, American Indian, and subjects of unknown race/ethnicity. Other demographic variables are age, employment, region of country, employment. Measurements and definitions of height, income, wages as well as other variables may vary in the vast literature and research conducted by economists, social scientists, psychologists, epidemiologists and others. Therefore, definitions in the WHI OS Data Set questionnaire for the major variables analyzed are shown as follows:

- Height, in inches at age 18 or tallest adult height.
- Income “total family income (before taxes) from all sources within your household in the last year” Income is coded in 9 categories: 1) less than $10,000 (4.5%), 2) $10,000–19,999 (11.7%), 3) $20,000–34,999 (23.3%), 4) $35,000–49,999 (20.1%), 5) $50,000–74,999 (20.2%), 6) $75,000–99,999 (9,4%), 7) $100, 000–149,999 (6.8%), 8) $150,000 or more (3.9%); and 9) “Don't know” (3%) and a category, missing (4%). The mode is in the $20,000–34,000 category, the median in the $35,000–49,999 category, interpolated median about $43,000. The eight categories, excluding missing and “Don't know” were condensed to 5—1) less than $20,000 (16.16%), 2) $20,000–34,999 (23.31%), 3) $35,000–74,999 (40.24%), 4) $75,0000–99,999 (9.43%), 5) $100,000 or more (10.86%).

1. Education: 1) Didn't go to school (.09%), 2) Grade school (1–4 years) (.38%), 3) Grade school (5–8 years) (1.20%) 4) Some high school (9–11 years) (3.51%), 5) High school diploma or GED (16.15%). 6) Vocational or Training School (9.74%), 7) Some college or Associate Degree (26.49%), 8) College graduate or Baccalaureate Degree (11.39%). 9) Some Postgraduate or professional (11.76%), 10) Master's degree (15.73%), 11) Doctoral Degree (Ph.D., M.D., J.D., etc.) (2.76%), Missing (0.79%). Condensed into 3 categories: 1) less than high school (22.12%). 2) high school to some college (47.63%) 3) college graduate or more (30.36%).
2. General health—“In general, would you say your health is—on a five point scale: 1) excellent', 17.7%, 2) very good, 40.2%, 3) good, 31.7%, 4) fair, 8.8%, 5) poor, 0.9%), ‘missing’ 0.7%.”
3. “Likelihood of Depression”—scaled from 0 to 100—higher more likelihood. Likelihood of depression, a highly skewed continuous variable was dichotomized at less than or equal to the median (0.0073)/greater than the median.
4. “Religion gives strength and comfort”—three categories–none 12.5%, a little 24.0%, a great deal 63.0%, missing, 0.5%.
5. “Attend clubs, lodges, etc.”—6 categories—1) not at all in the past month, 43.9%; 2) once in the past month; 3) 2 or 3 times in the past month; 4) once a week 8.1%; 5} 2 or 6 times a week 5.6%; 6) every day 0.1%; missing 1.4%; condensed—none (43.89%), monthly (40.91%), weekly or more (13.84%).
6. Main job—present job or past job held the longest. Defined as “Managerial, professional specialty (Executive, managerial, administrative, professional occupations. Job titles include teacher, guidance counselor, registered nurse, doctor, lawyer, accountant, architect, computer/systems analyst, personnel manager, sales manager, etc.) Missing, 4.7%” No–54.02%, Yes—41.23%.
7. Pain– Quality of life subscale on pain. PAIN ranges from 0 to 100 with a higher score indicating a more favorable health state. From the Rand 36-Item Health Survey (SF-36).
8. Satisfied with quality of life, analogous to Cantril's ladder, 0-Satisfied to 10-Dissatisfied.
9. Rate quality of life, analogous to Cantril's ladder, 0-worst, 10-Best. ‘Happy’: During the past four weeks ‘Have you been happy’. Six point scale 1 = All, 2 = Most, 3 = A good bit, 4 = Some, 5 = A little bit, 6 = None of the time. (From 36/37). This scale was reversed: All = 6, Most = 5, Good Bit = 4, Some = 3, Little = 2, None = 1.
10. ‘Emotional well-being’, ranging from 0 to 100 with a higher score indicating a more favorable health state. The source of the scale is the Rand 36-Item Health Survey (SF-36). Computed from Form 36/37, questions 76, 77, 78, 80, and 82. Source: Rand 36-Item Health Survey (SF-36). Quality of life subscale on emotional well-being ranges from 0 to 100 with a higher score indicating a more favorable health state.
11. ‘Social support’ is the sum of nine components. Scores range from 9 to 45, higher scores more support. The 9 components, each ranging from 1) None, 2) A little, 3) Some, 4) most, 5) All–of the time, are: Someone - a) ‘to listen when need to talk’, b) ‘to give good advice’; c) ‘who can take you to the doctor’, d) ‘to have a good time with’, e) ‘to help understand a problem when you need it’, f) ‘to help with daily chores if you are sick’, g) ‘to share your private worries’, h) ‘to do something fun with’, i) ‘to love you and make you feel wanted’.

### Statistical methods

Descriptive statistics (means and standard deviations), chi-square analyses for categorical data, linear regression and multivariable analyses of covariance (GLM) were carried out. Multivariable GLM analyses yielded means, standard errors, and p-values controlling for covariates, and pair-wise p-values by class.

## Results

Descriptive data from univariate analyses are in Table 1. The mean age for all women is 62.62 years; for Non-White, 62.32, for White 62.90, a significant difference, P<0.0001. Height in inches differs by race/ethnicity—Non-White 63.63, White 63.67, P = 0.033. Compared to Non-White women, White women's income was higher, P = 0.0128; self-reported general health was better, P = 0.0012; and fewer reported a great deal of strength and comfort from religion—63.6% vs., 62.9%, P = 0.0290. Subjective well-being and demographic variables did not differ. (Table 1).

**Table 1:** Descriptive Data All Women and by Non-White/White.

Univariate Means		Means					Percentages		
Continuous Variables	All	Non-White	White	P-Value#	Categorical Variables	All	Non-White	White	P-Value#
**Age**	63.62	**62.23**	**63.90**	**<0.0001**	**Income**				
**Height Inches**	63.67	**63.63**	**63.67**	**0.0330**	<$20k-	16.16	16.85	16.02	
**Happy (1–5)** *	4.55	4.53	4.55		$20k-	23.31	23.12	23.35	
**Emotional Well-being (0–100)**	78.57	78.38	78.61		$35k_	40.24	40.19	40.25	
**Satisfied with Life (11 Dissat-Sat)**	8.10	8.10	8.10		$75K-	9.43	15.87	9.41	
**Quality of Life (11 Worst-Best)**	8.25	8.25	8.25		$100k-	10.86	10.31	10.97	**0.0128**
**Social Support (9–45)**	35.92	35.87	35.93		**Education**				
**Pain Construct (0–100)** **	74.20	73.90	74.26		<High School	22.12	22.34	22.07	
**Likelihood of Depression (0–100)**	0.042	0.044	0.042		High Sch–Some College	47.63	47.72	47.61	
					College Grad or More	30.26	29.94	30.32	
					**Health–Exc/VeryGood** ∧	57.92	**56.94**	**58.12**	**0.0151**
					**Managerial/Professional Job** ∧∧	41.23	40.75	41.33	
					**Clubs**				
					None	43.89	43.85	43.90	
					Monthly	40.91	41.01	40.89	
					Weekly	13.84	13.81	13.84	
					**Strength/Religion**				
					None	12.51	11.86	12.64	
					A Little	24.01	24.01	24.00	
					A Great Deal	62.98	**63.60**	**62.86**	**0.0209**
					**Likelihood Depression**				
					None≤Median	55.38	55.43	55.37	
					Yes<Median	44.62	44.57	44.63	

* Parentheses show scale.

** Higher–Less Pain.

# Blank Not significant.

∧ vs.Good/Fair/Poor.

∧∧ vs. No Mang Job.

P-Values denote Non-White vs. White differences.

Univariate and multivariable covariance analyses for height as the outcome were carried out for the 93,676 participants into three groups a) all, b) Non-White and c) White women. Univariate means for height by demographic, behavioral and subjective well-being variables are in Table 2. Income and club attendance were significantly associated with height among all, Non-White and White women. However, in the two lowest income categories–<$20,000 and $20,000–$34,999–the height differences were greatest. Means for subjective well-being variables tended to be high among all women–in the top quintile, but they were not related to height.

**Table 2:** Mean Height in Inches.

	All			Non-White			White		
	Mean	Std. Dev.	P-value#	Mean	Std. Dev.	P-Value#	Mean	Std. Dev.	P-value#
**Variables**	63.67	2.49		**63.63**	2.49		**63.67**	2.49	
**Age**									
50–59	63.67	2.48		63.62	2.48		63.68	2.48	
60–69	63.66	2.48		63.65	2.52		63.67	2.48	
70–79	63.67	2.50		63.59	2.45		63.68	2.51	
**Income**									
<$20k	**63.63**	2.50	**0.0134** *	**63.53**	2.52	**0.0489** *	**63.65**	2.49	**0.0723** *
$ 20K-	**63.70**	2.47		**63.66**	2.48		**63.70**	2.47	
$35K-	63.67	2.49		63.64	2.49		63.68	2.49	
$75K-	63.68	2.49		63.66	2.41		63.69	2.51	
≥$100K	63.66	2.48		63.60	2.56		63.67	2.46	
**Education**									
<High School	63.67	2.48		63.62	2.50		63.68	2.47	
High Sch–Some College	63.67	2.48		63.64	2.48		63.67	2.49	
College Grad or More	63.66	2.50		63.61	2.52		63.67	2.49	
**Managerial/Professional Job**									
Missing	63.66	2.49		63.56	2.51		63.68	2.49	
No	**63.65**	2.48	**0.0723**	63.62	2.49		63.66	2.48	
Yes	**63.68**	2.49		63.65	2.50		63.69	2.49	
**Attend Club/Lodges/Groups**									
Missing	63.67	2.53		63.86	2.52		63.63	2.53	
None	**63.65**	2.49	**0.0015** **	**63.60**	2.50	**0.0050** **	**63.67**	2.48	**0.0272** **
Monthly	**63.66**	2.49	**0.0023** **	**63.61**	2.50	**0.0094** **	**63.67**	2.49	**0.0298** **
Weekly or more	**63.73**	2.48		**63.77**	2.48		**63.73**	2.48	
**Religion–Strength/Comfort**									
Missing	63.75	2.69		64.21	2.88		63.66	2.65	
None	**63.65**	2.49	**0.0843** ∧	63.67	2.50		**63.65**	2.49	**0.0398** ∧
A little	**63.70**	2.48		63.64	2.49		**63.71**	2.48	
A great deal	**63.65**	2.48	**0.0133** ***	63.64	2.49		**63.66**	2.48	**0.0175** ***
**General Health**									
Excellent/Very Good	63.67	2.48		**63.67**	2.48	**0.0058**	63.67	2.48	
Good/Fair/Poor	63.66	2.50		**63.56**	2.51		63.68	2.50	
**Happy**									
No	63.67	2.48		63.59	2.51		63.69	2.48	
Yes	63.67	2.49		63.64	2.48		63.67	2.49	
**Social Support–Median** *									
Above	63.67	2.49		63.61	2.49		63.68	2.49	
At or Below	63.67	2.48		63.66	2.50		63.67	2.48	
**Emotional Well-being–Median** *									
Above	63.67	2.49		63.59	2.50		63.68	2.49	
At or Below	63.67	2.48		63.66	2.48		63.67	2.48	
**Satisfaction with Life–Median** *									
Above	63.67	2.49		63.64	2.48		63.68	2.49	
At or Below	63.66	2.49		63.61	2.51		63.67	2.48	
**Quality of Life–Median** *									
Above	63.68	2.49		63.64	2.49		63.68	2.49	
At or Below	63.66	2.49		63.62	2.49		63.67	2.48	

# **Blank Not Significant.**

* $20k- taller then <$20k.

∧ **‘A little taller than ‘None’.**

** ‘Weekly taller than ‘Non’ and ‘Monthly’.

*** ‘A Little’ taller than ‘A great deal’.

Univariate Covariance Analyses.

Multivariable analyses included height and seven covariates. Table 3 shows pair-wise P-values as follows: 1) income—all, <$20 vs. $20k- P = 0.020; 2) education—none significant; 3) job—all women P = 0.0296, Non-White NS, White, P = 0.0360; 4) clubs—all, Non-White, White with weekly attendance were taller than none or monthly—for all, P = 0.0005 and P = 0.0039; Non-White, P = 0.0031 and 0.0201; White, P = 0.0137 and 0.0357; 5) religion—all and White women reporting ‘a little’ vs. ‘none’, and ‘a little’ vs. ‘a great deal’ were taller—all P = 0.0522 and P = 0.0039, White P = 0.0418 and P = 0.0130, Non-White NS; 6) general health–White women NS, Non-White women with excellent very good health were taller, P = 0.0116; 7). Taller women had a lower BMI; P<0.0001. Notably, results from univariate covariance analyses (Table 2) and multivariable covariance analyses (Table 3) show minor differences. Table 4 shows full results of the GLM multivariable covariance analyses for a) all women, b) Non-White women and c) White women. Height and subjective well-being—happiness, emotional well-being, satisfaction with life, quality of life, social support, general health and likelihood of depression—dichotomized at the median were not associated; with the exception, general health among Non-White women. (Table 5).

**Table 3:** Multivariable Covariance Analyses – Mean Heights.

	Pair Wise Comparisons		
	All Women		
	Mean Height	P-values	
**0 Non-White/White**			
**Non-White**	**63.669**	**0.0164**	
**White**	**63.724**		
**1 Income 1–5**		**1 vs 2**	
1 <$20k	**63.668**	**0.0210**	
2 $ 20K-	**63.732**		
3 $35K-	63.701		
4 $75K-	63.709		
5 ≥$100K	63.687		
**2 Education 1–3**		**NS**	
1 <High School	63.713		
2 High School–Some College	63.702		
3 College Graduate or More	63.683		
**3 Managerial/Professional Job**		**0.0296**	
No	**63.678**		
Yes	**63.724**		
**4 Attend Club/Groups**		**None vs. Weekly**	**Monthly vs Weekly**
None	**63.678**	**0.0005**	**0.0039**
Monthly	**63.693**		
Weekly	**63.770**		
**5 Strength/Comfort Religion**		**None vs Little**	**Little vs Great Deal**
None	63.673	**0.0524**	**0.0074**
A Little	**63.730**		
A Great Deal	63.676		
**6 General Health**		**NS**	
Good/Fair/Poor	63.657		
Excellent/Very Good	63.668		
**7 BMI Quartiles** *		**<0.0001**	
1	**63.952**		
2	**63.758**		
3	**63.619**		
4	**63.467**		

	Non-White			White		
	Mean Height	P-values		Mean Height	P-values	
**1 Income 1–5**		**NS**			**NS**	
1 <$20k	63.772			63.666		
2 $ 20K-	63.892			63.718		
3 $35K-	63.870			63.685		
4 $75K-	63.889			63.691		
5 ≥$100K	63.841			63.675		
**2 Education 1–3**		**NS**			**NS**	
1 <High School	63.875			63.699		
2 High School–Some College	63.861			63.688		
3 College Graduate or More	63.822			63.674		
**3 Managerial/Professional Job**						
No	63.878	**NS**		63.657	**0.0360**	
Yes	63.910			63.705		
**4 Attend Club/Groups**		**None vs Weekly**	**Monthly vs Weekly**		**None vs. Weekly**	**Monthly vs Weekly**
None	**63.793**	**0.0031**	**0.0201**	**63.675**	**0.0137**	**0.0357**
Monthly	**63.833**			**63.685**		
Weekly	**63.985**			**63.745**		
**5 Strength/Comfort Religion**		**NS**			**None vs Little**	**Little vs Great Deal**
None	63.813			63.664	**0.0418**	**0.0130**
A Little	63.826			**63.730**		
A Great Deal	63.779			63.675		
**6 General Health**		**0.0116**			**NS**	
Good/Fair/Poor	**63.594**			63.690		
Excellent/Very Good	**63.702**			63.681		
**7 BMI Quartiles** *		**<0.0001**			**<0.0001**	
1	**64.095**			**63.942**		
2	**63.903**			**63.748**		
3	**63.756**			**63.611**		
4	**63.656**			**63.448**		

* Significant Trend P<0.0001 Lowest BMI Highest Height.

**Table 4:** Results of Multivariable Covariance Analyses–Outcome Height—a: All Women, b: Non-White Women, c: White Women.

a: All Women	Class	Levels	Values				Mean Height	Std Error			P- values		
**0 Non-White/White 0/1**	**1**	2	0 1			**0 Non-White/White**			**0**	**1**			
**1 Income 1–5**	**2**	5	1 2 3 4 5			0 Non-White	63.6720	0.0453		**0.0168**			
**2 Education 1–3**	**3**	3	1 2 3			1 White	63.7264	0.0413					
**3 Managerial/Professional Job**	**4**	3	0 1 2			**1 Income 1–5**			**1**	**2**	**3**	**4**	**5**
**4 Attend Clubs/Groups**	**5**	4	0 1 2 3			1 <$20k	63.6677	0.0457		**0.0210**	0.2060	0.2535	0.5887
**5 Strength/Comfort Religion**	**6**	4	0 1 2 3			2 $ 20K-	63.7318	0.0443	0.0210		0.1662	0.4977	0.1606
6 General Health*	**7**	3	1 2 3			3 $35K-	63.7007	0.0430	0.2060	0.1662		0.7859	0.6325
**7 BMI Quartiles**	**8**	4	1 2 3 4			4 $75K-	63.7091	0.0495	0.2535	0.4977	0.7859		0.5540
	**Source**	**DF**	**SumSq**	**Mean Sq**	**F Value**	5 ≥$100K	63.6867	0.0487	0.5887	0.1606	0.6325	0.5540	
	**Model**	20	2969.786	148.4893	24.17	**2 Education 1–3**			**1**	**2**	**3**		
	**Error**	85128	522994.2884	6.1436		1 <High School	63.7128	0.0454		0.6351	0.2963		
	**CorrTot**	85148	525964.0745			2 Hi Schl–Some Coll	63.7019	0.0428	0.6351		0.3882		
	**R Sq**	**Coeff Var**	**RtMSE**	**SumSq**		3 Coll Grad or More	63.6829	0.0443	0.2963	0.3882			
	0.005646	3.892905	2.478633	63.67053		**3 Manag/Prof Job**			**1**	**2**	**3**		
**Source**	**DF**	**Type I SS**	**Mean Sq**	**F Value**	**Pr>F**	0 Missing	63.6957	0.0564		0.6812	0.5264		
**0 Non-White/White 0/1**	1	35.484644	35.484644	5.78	**0.0162**	1 No	63.6783	0.0412	0.6812		0.0296		
**1 Income 1–5**	4	40.026382	10.006595	1.63	0.1639	2 Yes	63.7236	0.0419	0.5264	**0.0296**			
**2 Education 1–3**	2	0.009905	0.004952	0	0.9992	**4 Clubs**			**1**	**2**	**3**	**4**	
**3 Managerial/Professional Job**	2	27.73049	13.865245	2.26	**0.1047**	0 Missing	63.6556	0.0756		0.7840	0.6511	0.1811	
**4 Attend Clubs/Groups**	3	70.745207	23.581736	3.84	**0.0092**	1 None	63.6784	0.0469	0.7840		0.4238	**0.0005**	
**5 Strength/Comfort Religion**	3	47.895507	15.965169	2.6	**0.050**	2 Monthly	63.6932	0.0471	0.6511	0.4238		**0.0039**	
6 General Health*	2	8.486091	4.243046	0.69	0.5013	3 Weekly or more	63.7695	0.0507	0.1811	0.0005	0.0039		
**7 BMI Quartiles**	3	2739.40779	913.135932	148.63	<.0001	**5 Religion**			**1**	**2**	**3**	**4**	
**Source**	**DF**	**Type III SS**	**Mean Sq**	**F Value**	**Pr>F**	0 Missing	63.7178	0.1274		0.7535	0.9294	0.7653	
**0 Non-White/White 0/1**	1	35.112271	35.112271	5.72	**0.0168**	1 None	63.6729	0.0490	0.7535		**0.0524**	0.9172	
**1 Income 1–5**	4	36.17002	9.042505	1.47	0.2077	2 A Little	63.7304	0.0459	0.9294	0.0524		0.0074	
**2 Education 1–3**	2	7.18059	3.590295	0.58	0.5574	3 A Great Deal	63.6756	0.0436	0.7653	0.9172	**0.0074**		
**3 Managerial/Professional Job**	2	29.096621	14.54831	2.37	**0.0937**	**6 General Health**			**1**	**2**	**3**		
**4 Attend Club/Groups**	3	76.594946	25.531649	4.16	**0.0059**	1 G/F/P	63.6570	0.0406		0.5293	0.3246		
**5 Strength/comfort Religion**	3	47.462193	15.820731	2.58	**0.052**	2 Exc/VG	63.6679	0.0399	0.5293		0.3717		
6 General Health*	2	7.817281	3.90864	0.64	0.5293	3 Missing	63.7727	0.1063	0.3246	0.3717			
**7 BMI Quartiles**	3	2739.40779	913.135932	148.63	<.0001	**7 BMI Quartiles**			**1**	**2**	**3**	4	
						1	63.9523	0.0443		<0.0001	<0.0001	<0.0001	
						2	63.7583	0.0444	<0.0001		<0.0001	<0.0001	
						3	63.6190	0.0444	<0.0001	<0.0001		<0.0001	
						4	63.4671	0.0442	<0.0001	<0.0001	<0.0001		

b: Non-White	Class	Levels	Values					Mean Height	Std Error			P- values		
**1 Income 1–5**	**1**	5	1 2 3 4 5				**1 Income 1–5**			1	2	3	4	5
**2 Education 1–3**	**2**	3	1 2 3				1 <$20k	63.7721	0.1073		**0.0758**	0.1253	0.1848	0.4326
**3 Managerial/Professional Job**	**3**	3	0 1 2				2 $ 20K-	63.8922	0.1043	0.0758		0.6839	0.9706	
**4 Attend Clubs/Groups**	**4**	4	0 1 2 3				3 $35K-	63.8697	0.1013	0.1253	0.6839		0.7955	0.6917
**5 Strength/Comfort Religion**	**5**	4	0 1 2 3				4 $75K-	63.8892	0.1171	0.1848	0.9706	0.7955		0.6038
6 General Health*	**6**	3	1 2 3				5 ≥$100K	63.8405	0.1160	0.4326	0.5207	0.6917	0.6038	
**7 BMI Quartiles**	**7**	4	1 2 3 4				**2 Education 1–3**			**1**	**2**	**3**	**4**	
	**Source**	**DF**	**SumSq**	**MeanSq**	**F Value**	**P-value**	1 <High School	63.87542	0.10680		0.7945	0.4484		
	**Model**	19	590.0410	31.0548	5.02	<.0001	2 Hi Schl–Some Coll	63.86066	0.10008	0.7945		0.4747		
	**Error**	14200	87827.4650	6.1850			3 Coll Grad or More	63.82214	0.10458	0.4484	0.4747			
	**CorrTot**	14219	88417.5061				**3 Manag/Prof Job**			**1**	**2**	**3**		
	**R Sq**	**Coeff Var**	**RtMSE**	**SumSq**			0 Missing	63.76961	0.13465		0.2954	0.1919		
	0.006673	3.9088	2.4870	63.6249			1 No	63.87821	0.09654	0.2954		0.53		
	**Source**	**DF**	**Type I**	**MeanSq**	**F Value**	**Pr>F**	2 Yes	63.91039	0.09782	0.1919	0.53			
**1 Income 1–5**	**1**	4	30.8849	7.7212	1.25	0.288	**4 Clubs**			**1**	**2**	**3**	**4**	
**2 Education 1–3**	**2**	2	2.2607	1.1304	0.18	0.833	0 Missing	63.8000	0.1872		0.973	0.876	0.3996	
**3 Managerial/Professional Job**	**3**	2	8.9379	4.4689	0.72	0.4855	1 None	63.7928	0.1131	0.973		0.3712	**0.0031**	
**4 Attend Clubs/Groups**	**4**	3	62.2094	20.7365	3.35	**0.0181**	2 Monthly	63.8335	0.1137	0.876	0.3712		**0.0201**	
**5 Strength/Comfort Religion**	**5**	3	21.8405	7.2802	1.18	0.31680	3 Weekly or more	63.9847	0.1228	0.3996	0.0031	0.0201		
6 General Health*	**6**	2	72.8989	36.4494	5.89	**0.0028**	**5 Religion**			**1**	**2**	**3**	**4**	
**7 BMI Quartiles**	**7**	3	391.0087	130.3362	21.07	<.0001	0 Missing	63.9935	0.3136		0.6129	0.6371	0.5428	
	**Source**	**DF**	**Type III**	**MeanSq**	**F Value**	**Pr>F**	1 None	63.8126	0.1192	0.6129		0.8534	0.6092	
**1 Income 1–5**	**1**	4	22.8336	5.7084	0.92	0.4494	2 A Little	63.8263	0.1104	0.6371	0.8534		0.3414	
**2 Education 1–3**	**2**	2	4.1767	2.0883	0.34	0.7135	3 A Great Deal	63.7786	0.1054	0.5428	0.6092	0.3414		
**3 Managerial/Professional Job**	**3**	2	10.8563	5.4282	0.88	0.4158	**6 General Health**			**1**	**2**	**3**		
**4 Attend Clubs/Groups**	**4**	3	54.5662	18.1887	2.94	**0.0318**	1 G/F/P	**63.5944**	0.0972		**0.0116**	0.0195		
**5 Strength/Comfort Religion**	**5**	3	8.1560	2.7187	0.44	0.7247	2 Exc/VG	**63.7019**	0.0955	0.0116		0.0498		
6 General Health*	**6**	2	67.6623	33.8311	5.47	**0.0042**	3 Missing	64.2619	0.2551	0.0195	0.0498			
**7 BMI Quartiles**	**7**	3	391.0087	130.3362	21.07	<.0001	**7 BMI Quartiles**			**1**	**2**	**3**	4	
							1	64.0951	0.1036		<0.0001	<0.0001	<0.0001	
							2	63.9033	0.1044	<0.0001		<0.0001	<0.0001	
							3	63.7562	0.1047	<0.0001	<0.0001		<0.0001	
							4	63.6563	0.1042	<0.0001	<0.0001	<0.0001		

C: White	Class	Levels	Values					Mean Height	Std Error			P- values		
**1 Income 1–5**	**1**	5	1 2 3 4 5				**1 Income 1–5**			**1**	**2**	**3**	**4**	**5**
**2 Education 1–3**	**2**	3	1 2 3				1 <$20k	63.6657	0.0497		**0.0860**	0.4905	0.5170	0.8138
**3 Managerial/Professional Job**	**3**	3	0 1 2				2 $ 20K-	63.7179	0.0481	0.0860		0.1850	0.4694	0.2174
**4 Attend Clubs/Groups**	**4**	4	0 1 2 3				3 $35K-	63.6854	0.0466	0.4905	0.1850		0.8586	0.7380
**5 Strength/Comfort Religion**	**5**	4	0 1 2 3				4 $75K-	63.6914	0.0539	0.5170	0.4694	0.8586		0.6861
6 General Health*	**6**	3	1 2 3				5 ≥$100K	63.6747	0.0529	0.8138	0.2174	0.7380	0.6861	
**7 BMI Quartiles**	**7**	4	1 2 3 4				**2 Education 1–3**			**1**	**2**	**3**		
	**Source**	**DF**	**SumSq**	**MeanSq**	**F Value**	**P-value**	1 <High School	63.6992	0.0494		0.6616	0.4131		
	**Model**	19	2478.186	130.431	21.26	<.0001	2 Hi Schl–Some Coll	63.6882	0.0465	0.6616		0.5435		
	**Error**	70909	435032.898	6.135			3 Coll Grad or More	63.6736	0.0480	0.4131	0.5435			
	**CorrTot**	70928	437511.084				**3 Manag/Prof Job**			**1**	**2**	**3**		
	**R Sq**	**Coeff Var**	**RtMSE**	**SumSq**			0 Missing	63.6992	0.0615		0.3648	0.9078		
	0.005664	3.88964	2.4769	63.6797			1 No	**63.6570**	0.0447	0.3648		0.0360		
	**Source**	**DF**	**Type I**	**MeanSq**	**F Value**	**Pr>F**	2 Yes	**63.7048**	0.0454	0.9078	**0.0360**			
**1 Income 1–5**	**1**	4	21.1670	5.2918	0.86	0.4855	**4 Clubs**			**1**	**2**	**3**	4	
**2 Education 1–3**	**2**	2	0.5972	0.2986	0.05	0.9525	0 Missing	63.6433	0.0822		0.7288	0.6465	0.2695	
**3 Managerial/Professional Job**	**3**	2	28.0657	14.0329	2.29	0.1015	1 None	63.6746	0.0508	0.7288		0.6184	**0.0137**	
**4 Attend Clubs/Groups**	**4**	3	36.9570	12.3190	2.01	0.1105	2 Monthly	63.6847	0.0510	0.6465	0.6184		**0.0357**	
**5 Strength/Comfort Religion**	**5**	3	42.8023	14.2674	2.33	**0.0727**	3 Weekly or more	63.7455	0.0550	0.2695	0.0137	0.0357		
6 General Health*	**6**	2	0.8823	0.4412	0.07	0.9306	**5 Religion**			**1**	**2**	**3**	4	
**7 BMI Quartiles**	**7**	3	2347.7145	782.5715	127.56	<.0001	0 Missing	63.6786	0.1392		0.9277	0.739	0.9794	
	**Source**	**DF**	**Type III**	**MeanSq**	**F Value**	**Pr>F**	1 None	63.6645	0.0530	0.9277		**0.0418**	0.7236	
**1 Income 1–5**	**1**	4	21.9645	5.4911	0.9	0.4658	2 A Little	**63.7303**	0.0497	0.739	0.0418		0.0130	
**2 Education 1–3**	**2**	2	4.2149	2.1074	0.34	0.7093	3 A Great Deal	63.6747	0.0471	0.9794	0.7236	**0.0130**		
**3 Managerial/Professional Job**	**3**	2	28.8171	14.4086	2.35	**0.0955**	**6 General Health**			**1**	**2**	**3**		
**4 Attend Clubs/Groups**	**4**	3	39.7157	13.2386	2.16	**0.0907**	1 G/F/P	63.6903	0.0437		**0.0116**	0.0195		
**5 Strength/Comfort Religion**	**5**	3	43.1498	14.3833	2.34	**0.0709**	2 Exc/VG	63.6814	0.0429	0.0116		0.0498		
6 General Health*	**6**	2	1.3257	0.6629	0.11	0.8976	3 Missing	63.6893	0.1167	0.0195	0.0498			
**7 BMI Quartiles**	**7**	3	2347.7145	782.5715	127.56	<.0001	**BMI Quartiles**			**1**	**2**	**3**	4	
							1	63.9416	0.0482		<0.0001	<0.0001	<0.0001	
							2	63.7480	0.0481	<0.0001		<0.0001	<0.0001	
							3	63.6105	0.0482	<0.0001	<0.0001		<0.0001	
							4	63.4479	0.0480	<0.0001	<0.0001	<0.0001		

**General Health–Good/Fair/Poor vs Excellent Very Good.**

Note: Missing data included in Multivariable Analyses–for *Job, Club, Religion, Health (less than 1% for these variables).

**Table 5:** Height and Subjective Well-Being Variables.

		All	P-value *	Non-White	P-value *	White	P-value *
**Happiness**	**≤Median**	63.670	0.9734	63.586	**0.0318**	63.687	0.3905
	**>Median**	63.665		63.643		63.670	
	**Missing**	63.666		64.156	∧	63.560	
**Emotional Well-Being**	**≤Median**	63.664	0.8051	63.588	0.0594	63.680	0.8429
	**>Median**	63.668		63.659		63.669	
	**Missing**	63.708		63.874		63.672	
**Satisfaction with Life**	**≤Median**	63.671	0.5363	63.636	0.0582	63.678	0.9280
	**>Median**	63.661		63.612		63.671	
	**Missing**	63.755		64.160	∧	63.674	
**Quality of Life**	**≤Median**	63.675	0.2192	63.635	**0.0200**	63.683	0.7529
	**>Median**	63.663		63.619		63.672	
	**Missing**	63.818		64.250	∧	63.727	
**Social support**	**≤Median**	63.668	0.5343	63.607	0.2914	63.607	0.6522
	**>Median**	63.669		63.658		63.658	
	**Missing**	63.613		63.520		63.520	
**General Health**	**≤Median**	63.658	0.3236	63.559	**0.0004**	63.679	0.9144
	**>Median**	63.671		63.671		63.671	
	**Missing**	63.792		64.296	∧∧	63.686	
**Likelihood of Depression**	**≤Median**	63.657	0.5345	63.616	0.7771	63.666	0.3590
	**>Median**	63.675		63.640		63.682	
	**Missing**	63.651		63.581		63.667	0.6496

* P-values <0.05 Bold.

∧ Missing differs from <Median and >Median.

∧∧ <Median and >Median Differ, Missing Differs from <Median and >Median.

Income and education as predictors of subjective well-being, club attendance and religion revealed both congruencies and differences among Non-White and White women. Among White women, income and the subjective well-being variables—happiness, emotional well-being, happiness, satisfaction with life, quality of life and social support—and general health were significantly associated. These variables were also associated with education, with the exception of satisfaction with life. In contrast, Non-White women's subjective well-being variables—emotional well-being, happiness, and satisfaction with life—were not associated with income except for quality of life, P = 0.0095 and social support, P = 0.0007. Associations with education were significant for variables: happiness, emotional well-being and quality of life; satisfaction with life, but not significant for social support. (Table 6) An additional finding of interest is that measures of the likelihood of depression, unlike general health, showed no disparities by Non-White/White and no associations with height, (Tables 2 and 3) with income, and with education. (Table 6). ‘Strength and comfort from religion’—‘a great deal’–was associated with depression and the subjective well-being variables. Those with ‘a great deal’ had the highest values (means) from the subjective well-being variables. In contrast, those with ‘a great deal’ had poorer general health. (Table 7). Interestingly, income and education were associated with religion among White women. Those with higher income and with higher education were more likely to report ‘none’ and less likely to report ‘a great deal’ (Chi-square P<0.0001). Among Non-White religion and income and religion and education were not significantly associated. (Table 8).

**Table 6:** Subjective Well-Being Means by Income and Education.

Row 1 Non-White		Income						Education			
Row 2 White		<$20K	$20K-	$35K-	$75K-	≥$100K	P-Value	<High School	High School- Some College	College Grad or More	P-Value
**Happy**											
**1**		4.522	4.536	4.533	4.513	4.567	0.6584	4.491	4.545	4.541	**0.0299**
**2**		4.516	4.543	4.557	4.549	4.567	**0.0019**	4.531	4.554	4.552	**0.0501**
**Emotional Well-Being**											
**1**		78.012	78.356	78.462	78.770	78.512	0.6150	77.649	78.708	78.408	**0.0027**
**2**		78.059	78.635	78.741	78.576	78.781	**0.0006**	78.315	78.660	78.736	**0.0113**
**Satisfaction with Life**											
**1**		8.030	8.111	8.105	8.083	8.153	0.3637	7.997	8.124	8.126	0.3638
**2**		8.043	8.084	8.103	8.120	8.167	**0.0003**	8.089	8.107	8.091	0.4675
**Quality of Life**											
**1**		8.149	8.248	8.262	8.279	8.303	**0.0095**	8.164	8.266	8.285	**0.0008**
**2**		8.191	8.247	8.259	8.283	8.303	**<0.0001**	8.233	8.263	8.253	**0.0169**
	**Social Support**										
**1**		35.299	35.888	36.004	35.797	36.332	**0.0007**	35.673	35.906	35.969	0.2252
**2**		35.531	35.753	36.000	36.139	36.294	**<0.0001**	35.858	35.933	35.961	0.4196
**General Health** *											
**1**		2.425	2.381	2.345	2.325	2.357	**0.0018**	2.407	2.361	2.347	**<0.0001**
**2**		2.394	2.351	2.336	2.312	2.293	**<0.0001**	2.365	2.341	2.325	**0.0097**
**Likelihood of Depression** **											
**1**		0.0482	0.0433	0.0432	0.0410	0.0462	0.4714	0.0462	0.0427	0.0455	0.4196
**2**		0.0438	0.0435	0.0411	0.0413	0.0413	0.1909	0.0424	0.0420	0.0422	0.9394

*Low values better health – 1 = Excellent-5 = Poor.

** Low values less likelihood.

**Table 7:** Subjective Well-Being Variables by Strength and Comfort from Religion.

Women	All	Non-White	White
	Means	Means	Means
**Happy**			
None	4.409	4.379	4.415
A Little	4.42	4.402	4.424
A Great Deal	**4.621**	**4.609**	**4.623**
**Emotional Well-Being**			
None	77.82	77.25	77.927
A Little	76.884	76.592	76.943
A Great Deal	**79.364**	**79.272**	**79.382**
**Satisfaction with Life**			
None	7.796	7.797	7.796
A Little	7.788	7.784	7.789
A Great Deal	**8.277**	**8.271**	**8.278**
**Quality of Life**			
**Life**			
None	7.796	8.056	8.05
A Little	7.788	8.023	8.016
A Great Deal	**8.277**	**8.37**	**8.385**
**Social Support**			
None	35.097	35.094	35.097
A Little	34.945	34.89	34.956
A Great Deal	36.456	**36.397**	**36.468**
**General Health** *			
None	**2.143**	**2.15**	**2.142**
A Little	2.316	2.31	2.317
A Great Deal	2.397	2.428	2.391
**Likelihood of Depression** **			
None	0.044	0.0452	0.0438
A Little	0.0474	0.0498	0.0469
A Great Deal	**0.0403**	**0.0421**	**0.0399**

*Low values Better. General Health 1 = Excellent–5 = Poor.

** Low values less likelihood.

N.B. P<0.0001 for all groups and variables except Non-White Likelihood of Depression–P = 0.0334.

**Table 8:** Strength and Comfort from Religion by Income and by Education for All, Non-White, White Women Percentages for None, A Little and A Great Deal.

	Income	All Women				Education	All Women	
	<$20k	$20k-	$35k	$75K	≥$100k	<High School	High School Some College	College Grad or More
**None**	11.72	12.37	12.5	13.54	13.68	11.76	12.36	13.30
**A Little**	23.37	23.46	24.25	24.19	25.01	24.06	23.9	24.12
**A Great Deal**	64.43	63.58	62.77	61.71	60.92	63.66	63.24	62.08
		Chi-square	P<0.0001				P<0.0001	

			Non-White			Non-White		
	<$20k	$20k-	$35k	$75K	≥$100k	<High School	High School Some College	College Grad or More
**None**	11.33	12.22	11.58	12.95	12.63	11.69	11.91	11.78
**A Little**	23.16	22.72	24.8	25.54	25.07	24.58	23.59	23.95
**A Great Deal**	64.89	64.37	63.23	61.00	61.63	63.33	63.87	63.73
		Chi-square	P = 0.1272				P = 0.6029	

			White			White		
	<$20k	$20k-	$35k	$75K	≥$100k	<High School	High School Some College	College Grad or More
**None**	11.80	12.4	12.69	13.66	13.88	11.78	12.46	13.57
**A Little**	23.42	23.61	24.14	23.92	25.00	23.95	23.97	24.10
**A Great Deal**	**64.34**	63.42	62.67	61.86	60.79	63.73	63.11	61.83
		Chi-square	P<0.0001				P<0.0001	

In sum, new findings from this study of US women, 49–79, are: a) taller Non-White and White women engaged in more frequently in social activities, e.g., such as club attendance; b) taller White women had reported significantly more ‘a little’ strength and comfort from religion compared to ‘none’ and compared to ‘a great deal’. Other major findings are: c) taller Non-White and Whites did not have higher incomes or more education; d) taller White women with present or past managerial/professional jobs; e) taller Non-White women had better general health.

## Discussion

A vast and global literature examines the relation of height with numerous factors, including, but not limited to psychological, social, economic, anthropologic, genetic, gender, environmental, ecologic, behavioral, nutritional, infection and other constructs. This study examined data from relatively healthy women ages 49–79, from a range of race/ethnic groups—dichotomized Non-white 17% and White 83% of the sample of 93,676 women. It focused on height and variables including income, education, general health, social activities, and subjective well-being. Two major findings emerge: 1) taller Non-White and White women engaged social activities, viz. attended clubs/lodge/groups, more frequently than those who did not attend or attended less frequently. Attendance at clubs is one among a variety of social activities. Notably, this finding is in accord with Persico et al. [21], who related social activities, such as athletics, to height and wages–one of the few papers to analyze social activities.

2) Strength and comfort from religion was associated not only with height, but also with subjective well-being, general health, income and education. (Tables 1—4, 7–8). The association of religion and income has been discussed by Barro and McCleary [30]; and religion and health have many citations in the medical literature [31]. However, to my knowledge, religion and height have not been investigated.

Occupation and height of men and women have been examined by many investigators [7], [10], [14], [19], [21], as well as others. In particular, the paper of Case and Paxon, based on data from cohort (longitudinal) studies, concluded that taller adults select into occupations that have higher cognitive skill requirements and lower physical skill demands [7]. Case, Paxon and Islam confirm these results using longitudinal data from the BHPS (British Household Pane Survey [32]. In this study, taller White women had managerial/professional jobs, and taller Non-White women did not have managerial/professional jobs; but they had better general health–results consistent with the effects of genetics, environment, poverty, medical conditions, nutrition and cognitive skills.

However, height was not significantly associated with income nor with and education among both Non-white and White. This is in contrast to findings of Deaton and Arora, who analyzed the Analysis of the Gallup-Healthways Well-Being Index daily poll of the US population [10]. They reported “taller people lead better lives on average”–findings “almost entirely explained by the positive association between height and both income and education”. These differences in results may be accounted for by social and cultural factors in both White and Non-White women such as: a) in the U.S., women's incomes continue to lag those of men, for this reason, taller White women may lead better lives by virtue of their managerial/professional positions rather than by income or education; and b) Non-Whites with better health were taller; early environmental or genetics factors may have prevented some Non-Whites from reaching their full physical and mental development [7], [10]. It is noteworthy that, though not related to height, subjective well-being variables are significantly associated with income and education among White women. Hence, higher income and better educated women may lead better lives, but not because they are taller; findings that differ from Deaton and Arora [10].

A new area examined in this study is religiosity as measured as ‘strength and comfort from religion’ classified as ‘none’, ‘a little’ and ‘a great deal’. Overall results are the percentage of women reporting—12% ‘none’, 24% ‘a little’ and 63% ‘a great deal’, and 0.5% missing data. Analyses of this construct, both as a covariate and as a outcome, (to my knowledge has not examined in the literature on height), was related to height, as well as health, subjective well-being, income and education (Tables 2 and 3), Although measures and definitions of ‘religion/religiosity’ may differ among investigators, my findings on religion and income are in accord with Barro and McCleary [30]. Their findings reveal an overall pattern in which economic development is associated with less religiosity, measured by church attendance or religious beliefs. They conclude: “This pattern can be seen in simple relations between a measure of religiosity and per capita GDP, which we take as the basic indicator of economic development.” (Their future research plans include an assessment of the effects of religiosity on political and social variables, including democracy, the rule of law, fertility, and health. P 38). To my knowledge height and religion have not been investigated. Health and religion/religiosity are of increasing interest in the medical literature. November 18, 2013PUBMED search for ‘religion’ yielded 50054 hits. Koenig, Director, Center for Spirituality, Theology and Health at Duke University. “Reviews. Religion, Spirituality, and Health: the research and clinical implications” [31]. Interestingly, while weight is discussed, no mention of height is found in the text or among the 596 references.

Further research, suggested by my findings, on height and other factors are the following:

1. Occupation–indicated by the finding that taller White women had managerial/professional jobs presently or in the past. In the WHI data ‘managerial/professional job’ covers a range of occupations'. It is defined as “Managerial, professional specialty (Executive, managerial, administrative, professional occupations. Job titles include teacher, guidance counselor, registered nurse, doctor, lawyer, accountant, architect, computer/systems analyst, personnel manager, sales manager, etc.)”. To understand better the association of height and the components of ‘managerial/professional specialty need more detailed classifications.
2. Social activities—here denoted by attendance at clubs/lodges/groups—a construct significantly associated with height among Non-White and White. What constitutes social activities and how to measure them needs further work.
3. ‘Strength and comfort from religion’, and important construct in this study, was associated with height, income, education and health. Women who reported ‘a little’ vs. ‘none’ or vs. ‘a great deal’ were taller, had higher incomes and better education, but those with ‘none’ had better health. Importantly, as far as I am aware, religion/religiosity and height have not been previously examined. Replication and validation in other groups are suggested.

A possible limitation of this study is that the data are from a cross-section observational study, which may not be sufficient for analyzing changes over time or causal inference. The strengths of this study are the large sample size and reliability and validity of the questionnaire.

In conclusion, among relatively healthy U.S. women, 17% Non-White and 83% White, ages 49–79, height and income, and height and education, were not associated. However, taller White women had better jobs, and taller Non-White had better health. In addition, two new results emerged—first, taller Non-White and White women attended clubs/groups more frequently. Second, taller women reported ‘a little’ comfort from religion (vs. ‘none’ and vs. ‘a great deal’)–they add to the vast literature on height and its relation with human behavior and with well-being. Whether these findings are generalizable globally to diverse populations and a range of demographics– including age, gender, culture, socioeconomics, psychosocial, among others–raise important questions in search of answers.
